The article "Evaluation of Different Adhesive Resin Removal Methods after Debonding Ceramic Orthodontic Molar Tubes: A Scanning Electron Microscope Study" was published in 2022. Journal: Scanning.

# Evaluation of Different Adhesive Resin Removal Methods after Debonding Ceramic Orthodontic Molar Tubes: A Scanning Electron Microscope Study

**DOI:** 10.1155/2022/4853035

**Published:** 2022-11-16

**Authors:** Zeynep Atmaca, Mutahhar Ulusoy, Cagri Ulusoy

**Affiliations:** ^1^Gazi University Faculty of Dentistry, Department of Orthodontics, Ankara, Turkey; ^2^Faculty of Dentistry of Near East University, Department of Prosthodontics, Nicosia, Cyprus

## Abstract

**Objectives:**

To evaluate and compare the impacts, bond strength, residual adhesive, and time invested on the enamel surface after debonding of recently introduced ceramic buccal molar tubes with different systems.

**Materials and Methods:**

Ceramic molar tubes were bonded to fifty-four maxillary molar teeth, and a shear bond strength (SBS) test was performed. The adhesive remnant index (ARI) scores were recorded, and the samples were divided into two groups for adhesive removal with low-speed instruments: tungsten carbide bur or diamond-coated micropolisher point. The time to clean the enamel surfaces was also noted down for each tooth. The enamel surfaces were investigated with scanning electron microscope (SEM) after adhesives were cleaned. Shapiro-Wilk's, Kolmogorov-Smirnov's, and Student's independent *t* tests were used for statistical analysis.

**Results:**

The mean SBS value of the tested ceramic molar tubes was 9.78 ± 1.85 MPa, and the majority of the samples were scored as ARI 1 and ARI 2. No statistically significant difference between PoGo micropolisher and TCB was found in terms of time values for surface cleaning. The enamel surface characteristics of TCB for adhesive remnant removal resulted in a better enamel surface than the single-step diamond polisher when the samples were investigated by using SEM.

**Conclusions:**

Ceramic molar tubes may be an enamel-safe product for patients seeking for fully aesthetic orthodontic treatment, if used in carefully handled clinical conditions. One-step polishing systems utilised with low-speed instruments could be used confidentially for cleaning the resin remnants on enamel after orthodontic treatment.

## 1. Introduction

The rising number of adult patients questing for orthodontic treatment with less apparent equipment prompted the development of ceramic brackets in orthodontics three decades ago [1]. Ceramic brackets, notwithstanding their higher aesthetics, featured higher bond strength and weaker fracture toughness than metal brackets, creating issues in the course of debonding such as enamel tear outs, minor fractures, and cracks [2, 3].

The orthodontist's priority should be to preserve the enamel surface as much as possible to natural enamel without inflicting iatrogenic damage and with few enamel struc ture loss [4]. The rough surface of the enamel restricts adequate cleaning, which promotes plaque build-up, bacterial storage, and stain formation, degrading the aesthetic quality. Restoring enamel to its natural morphological characteristics is challenging [5]. A range of technical processes have been developed to achieve successful resin removal with the smallest level of enamel impairment possible after bracket debonding. One-step polishing systems and carbide burs are some examples of these methods [3–5].

The purpose of this research was to analyze and compare the impacts, residual adhesive, and time invested on the enamel surface after structural debonding of recently introduced ceramic buccal molar tubes with mainstream systems using a scanning electron microscope (SEM).

## 2. Materials and Methods

This study was approved by Gazi University Research Ethics (2020-561). The sample size calculations of the current study were decided according to the metaepidemiological study of Mheissen et al. [6] investigating 147 orthodontic trials which pointed out that 60.4% of the studies selected 80% for the power analysis. The sample size was estimated by power analysis considering a significance threshold of 0.05 and a power of 80% to identify substantial differences between the mean values of two groups. It revealed that a minimum of 25 samples were required for each group. Therefore, 27 samples per group, which makes a total of 54 samples for two groups, were gathered in order to conduct the study.

In this in vitro experiment, 54 first-molar permanent human maxillary teeth freshly extracted for periodontal concerns were collected and preserved in filtered water for four weeks at room temperature with 0.1% thymol crystals added. Molars that had (1) caries, (2) restorations, (3) obvious cracks, or (4) abnormalities were excluded from the study.

Each tooth was embedded in a cold-cured acrylic resin mold prior to the orthodontic bonding procedure. The teeth were oriented in the resin molds, so that the buccal surface was perpendicular to the bottom of the mold to align the bonded surface parallel to the test machine blade.

Fifty-four teeth were etched for 30 seconds with 37% orthophosphoric acid (3M ESPE, St. Paul, Minnesota, USA), washed for 10 seconds, and dried using oil-free compressed air. Only one practicing orthodontist placed the polycrystalline ceramic buccal tubes (Phantom Buccal Ceramic Tube, Gestenco International AB, Göteborg, Sweden) in their appropriate position on the crown and bonded them with Transbond XT primer and adhesive paste (3M/Unitek, Monrovia, California, USA) (Figure 1). Excess bonding was carefully removed, and the ceramic tubes were light-cured from their geometric center for three seconds using a LED curing unit (VALO Ortho Cordless, Ultradent GmbH, Cologne, Germany).

After bonding the molar tubes, all specimens were stored in distilled water at 37°C for 24 hours. The samples were then placed in a universal testing machine (Lloyd Instruments Ltd., Fareham, UK) for the shear bond strength (SBS) test. Molar tubes were subjected to the shear bond test using a 1 kg load cell and a velocity of 1 mm/min [7] (Figure 2). The force that resulted in the breakdown was measured in Newton and then translated to megapascal (MPa) by dividing the measured force values by the mean surface area in millimeters.

The quantity of adhesive residuals on teeth after the tubes were debonded was evaluated with naked eye using Artun and Bergland's [8] adhesive remnant index (ARI) methodology. The following are the parameters for this index system:

- Score 0: no adhesive left on the tooth
- Score 1: less than half of the remaining adhesive on the tooth
- Score 2: more than half of the remaining adhesive on the tooth
- Score 3: all adhesive remained on the tooth (sometimes with a distinct impression of the bracket mesh)

The tubes were randomly assigned to two groups after being removed from the enamel surface.

- Group 1: 8-fluted TCB with a working surface length of 4 mm (Hager & Meisinger GmbH, Neuss, Germany) by low-speed hand piece with air cooling (*n* = 27) (Figure 3(a))
- Group 2: diamond-coated PoGo micropolisher point (Dentsply Caulk, Milford DE, USA) by low-speed hand piece with air cooling (*n* = 27) (Figure 3(b))

The enamel surfaces were cleaned by the same experimenter in all samples under continuous air flow to ensure the visibility of the enamel surface, and the intervals were measured. After a 3 nm thick gold-palladium coating, the samples were analyzed using a scanning electron microscope (QUANTA 400F Field Emission SEM, Philips/FEI, Hillsboro, OR, USA) at a high resolution (1.2 nm).

The data obtained in this study were analyzed with the IBM SPSS 21 package program (IBM SPSS Statistics, New York, USA). Shapiro-Wilk's and/or Kolmogorov-Smirnov test was used for investigating the normal distribution of the variables. The significance level for the interpretation of the data was set at 0.05; if *p* < 0.05, it was determined that the variables did not come from a normal distribution. Based on the results of the data normality tests, Student's independent *t* test was used for two-group comparisons.

## 3. Results

According to the SBS test results, the mean value of the samples was 9.78 ± 1.85 MPa (minimum recorded value 6.11 MPa and maximum recorded value 13.92 MPa).

When the ARI scores were observed, most of the samples were scored as 1 and 2 (Table 1). No sample was recorded as ARI 3.

SEM images of the intact enamel surface and the base of the ceramic molar tube can be seen in Figures 4 and 5, respectively. The square-shaped molar tube had rounded corners, and the mesh base was composed of square-shaped holes. SEM analysis of enamel surfaces after the use of TCB and PoGo micropolisher systems is shown in Figure 6, and it was 7 and found similar to the characteristics of an intact tooth in Figure 4.

Using a TCB for adhesive remnant removal resulted in a better enamel surface (Figures 6(a) and 6(b)) than the adhesive remnant removal with single-step diamond polisher, PoGo, operated at low speed (Figures 7(a) and 7(b)). Cleaning the surface with PoGo showed minor scratches on the enamel surface.

In terms of time values, there was no statistically significant difference between the PoGo micropolisher and the TCB (*p* > 0.05) (Table 2 and Figure 8).

## 4. Discussion

Patients requesting invisible and aesthetic orthodontic treatment appliances for their treatments are increasing day by day; therefore, manufacturers are commonly offering new products to fulfill their demand. Although cosmetically popular ceramic brackets were introduced decades ago [1], ceramic molar tubes were recently introduced to generate a fully transparent and invisible appearance for the whole dental arch.

There are studies measuring the SBS of ceramic brackets [9, 10] and investigating different finishing methods after debonding, but no studies were conducted with the ceramic molar tubes to our knowledge. In this study, different rotary tools were used to remove residual adhesive after the ceramic tubes were separated from the enamel surface; the time spent was recorded, and the effects on the enamel surface were examined under SEM.

The fact that ceramic brackets have a higher SBS than metal brackets had been revealed in previous investigations [9, 11]. In vitro studies showed a wide range in variation for SBS values. Chung et al. [10] found the SBS values of ceramic brackets as 15.66 ± 7.05 MPa, and Olsen et al.'s [12] results were 10.56 ± 6.0 MPa, whereas Mirhashemi et al.'s [13] mean SBS values were 7.46 ± 1.4 MPa in their studies. In the present study, the mean SBS value for ceramic molar tubes was 9.78 ± 1.85 MPa which was harmonious with the previous works. Shear bond forces in Newtons were converted to MPa by dividing them with ceramic tube base area values, which were larger when compared with bracket base areas; therefore, our results were not as high as Chung et al. [10]. The variations in buccal side morphology of the tested teeth, bonding procedures, base area, properties of the orthodontic material, and accuracy in placing the blade of the machine in debonding test might be counted among the different results in the studies [10, 14, 15].

It must be remembered that gathering superior bond strength should not be the main objective of the clinician because debonding the appliances without giving any harm to enamel surface is the fundamental point. Although Reynolds [16] stated that the acceptable bond strength of orthodontic appliances for clinical practice should be between 5.88 and 7.85 MPa, Mizrahi and Smith [17] estimated the sufficient bond strength for orthodontic brackets in the range of 2.8 to 10 MPa. Retief [18] suggested that SBS values above 9.7 MPa could lead to enamel fractures; however, Forsberg and Hagberg's [19] findings showed that the risk of enamel damage starts about 30 MPa for some patients. The ceramic molar tubes in the present study have generated biocompatible SBS values which might be attributed to undercut mesh in their bases designed for easy debonding.

The SEM images were used not only to compare the enamel surfaces after two different adhesive removal techniques but also compare these images with the enamel surface of the intact tooth in the current study. The investigation of microstructure of the tube base, its possible effect on enamel cracks, and evaluation of adhesive remnants after debonding could be counted among the other benefits of SEM. The SEM images were taken after cleaning the surfaces either with TCB or PoGo micropolisher systems; therefore, adhesive remnants could not be located on enamel surfaces on any of the samples tested. Indeed, the main point of choosing SEM as a diagnostic tool for our study was to make the comparison of enamel surfaces after adhesive removal.

When the ARI data of the current study were evaluated, it was seen that the adhesive remained mostly on the ceramic tubes as expected. No samples were scored as ARI 3, maintaining a beneficial situation to reduce the time spent to clean the enamel surface. Although 15 teeth were scored as ARI 0, no cracks were detected when the enamel surfaces were evaluated with SEM. Based on our findings, it could be noted that the ceramic molar tubes did not cause damage to enamel surface as recommended by previous studies [2, 10].

The method selected to remove residual resin after debonding was reported to be critical in preventing enamel surface damage such as cracks in enamel, rougher enamel surface, enamel wear, overheating of the teeth, and pulpal damage [20]. However, it is also important to remove the residual adhesive in the shortest possible time for the patient and the clinician as well. No significantly different results between the adhesive removal protocols tested in the current study were obtained for the time spent to remove resin remnants from enamel surfaces. Less time might be spent for TCB group, if a high-speed rotary system was selected, but more damage to the enamel surface should be expected, similar to previous studies [21, 22].

Previous studies used various methods for cleaning the residual resin after removal of orthodontic attachments such as Er:YAG laser [20], hydrobrasion with rotary instruments [21], conventional carbide burs [23], tungsten carbide burs in different shapes [24], and adhesive removal discs [24]. Among all these methods, tungsten carbide burs were the most popular instruments in both low and high speed for residual adhesive removal [21]; therefore, we had chosen this tool for one of the protocols tested in the current study. Some studies revealed that their use on low-speed motors maintains better results for resin removal [22, 25]; hence, low-speed hand piece under air cooling was chosen for both TCB and PoGo groups in this research.

Except for some samples cleaned by using PoGo, both systems tested in the present study generated enamel surfaces similar to the intact tooth when the SEM images were compared. Our results might seem conflicting with the previous studies [24, 26] that found TCB causing enamel scarring, thus requiring multistep polishing. The tungsten carbide burs were used at low speed in the present study, which might be a reason for achieving results differentiating from the others that use TCB in high speed [26, 27].

PoGo single-step polisher was used on the enamel without any surface pretreatment and under continuous air flow without water as suggested in the previous studies [28, 29]. Although PoGo produced minor marks on enamel surface in some samples, this product had also maintained clean enamel surface consistent with previous studies [26, 30]. Application of pressure against enamel surface and selection of rotational speed during the cleaning process had been shown among the operator-dependent factors in a study investigating enamel surface after debonding [31]; therefore, better results may be obtained by experienced clinicians. Additionally, also saliva moistening [32], blood contamination [33], and the use of fluoridated pastes [7] have been shown among the factors that have influence on bond strength. These variables should also be evaluated in future SEM studies.

Most studies evaluating the removal of adhesive resins have been conducted in vitro, as in our study, eliminating some factors that could have affected bonding and debonding orthodontic instruments. Salivary hydration of teeth surfaces, treating enamel surfaces with fluoride products, and absence of ion exchange between saliva and teeth could be counted among these in vivo environmental factors that could not be easily mimicked in vitro. Both debonding and adhesive resin removal are operator-dependent procedures, and only one operator performed all the investigations in our study which could be counted as a serious limitation. Future research comparing more adhesive removal techniques in greater sample sizes is needed.

## 5. Conclusions

Taking into account the limitations of this in vitro study, the ceramic molar tubes may be an enamel-safe product for patients seeking for fully aesthetic orthodontic treatment, if used under carefully handled clinical conditions. The results of this research also indicated that one-step polishing systems used with low-speed instruments could be used confidentially to remove enamel resin remnants on enamel after orthodontic treatment.

## Figures and Tables

**Figure 1:** The polycrystalline ceramic orthodontic tube tested in the study.

**Figure 2:** Application of shear force produced by universal testing machine to orthodontic molar tubes.

**Figure 3:** (a) 8-fluted tungsten carbide bur (TCB). (b) Diamond-coated micropolisher point.

**Figure 4:** SEM image of intact tooth enamel surface.

**Figure 5:** SEM image of the base of ceramic molar tube.

**Figure 6:** (a) Enamel surface after removal of adhesive remnant using TCB under 50x magnification. (b) Image from the same region under 100x magnification.

**Figure 7:** (a) Enamel surface after removal of adhesive n using PoGo micropolisher under 50x magnification. Note the scratches on surface. (b) Image from the same region under 100x magnification.

**Figure 8:** Histogram showing adhesive remnant removal time in seconds of the tested materials.

**Table 1:** Adhesive remnant index (ARI) scores of the tested 54 samples. *n*: number of samples; PoGo: PoGo micropolisher; TCB: tungsten carbide bur.

ARI scores	0	1	2	3
PoGo (*n*: 27)	7	11	9	0
TCB (*n*: 27)	8	10	9	0

**Table 2:** Analysis result regarding the difference between groups in terms of duration values.

Groups	Time (seconds)						Independent *t* test	
	*n*	Mean	Median	Min	Max	SD	*t*	*p*
PoGo	27	21.66	20.25	13.20	36.85	6.32	-0.464	0.645
TCB	27	22.39	23.00	9.96	30.83	5.26		

## Data Availability

Data of this study is available on request. Please contact the corresponding author, Prof. Cagri Ulusoy, via the e-mail address mehmetcagri@gazi.edu.tr.
